This article has been retracted.

# A synthetic dsRNA, as a TLR3 pathwaysynergist, combined with sorafenib suppresses HCC in vitro and in vivo

**DOI:** 10.1186/1471-2407-13-527

**Published:** 2013-11-06

**Authors:** Yu-Yin Xu, Li Chen, Gui-Lan Wang, Jia-Ming Zhou, Yi-Xin Zhang, Yin-Ze Wei, Yuan-Yuan Zhu, Jing Qin

**Affiliations:** 1 Department of Pathological Anatomy, Nantong University, Nantong, China; 2 Department of Nephrology, Affiliated Hospital of Nantong University, Nantong, Jiangsu, China; 3 Department of Pathology, Affiliated Tumor Hospital, Nantong University, Nantong, China; 4 Biomics (Nantong) Co., Ltd, Nantong, China

**Keywords:** dsRNA, TLR3, NF-κB, sorafenib, HCC

## Abstract

**Background:**

Recent studies have demonstrated that synthetic dsRNAs may produce therapeutic effects in a target-independent manner through stimulation of the toll-like receptor-3 (TLR3)/interferon pathway; as a result, angiogenesis and proliferation of tumor cells are inhibited. Thus, this pathway may become a potential target of dsRNA in tumor suppression. In this study, we evaluated the role of synthetic dsRNA as a TLR3 synergist and by combining with sorafenib in anti-hepatocellular carcinoma (HCC) *in vitro* and *in vivo*.

**Methods:**

Four dsRNAs were designed and synthesized. One of them that was capable of activating TLR3 most effectively in human HCC cell line (HepG2.2.15) was selected as a TLR3 synergist (called BM-06). Subsequently, the expression of proteins relating to TLR3 signaling pathway, such as NF-κB, caspase 8 survivin, bcl-2 and PCNA affected by BM-06, sorafenib alone or in combination, was compared. The migration, proliferation and apoptosis of HepG2.2.15 cells were evaluated in presence of BM-06, sorafenib alone or in combination of both. The similar treatments were also applied in an SD rat primary HCC model.

**Results:**

qRT-PCR data showed that the expression of TLR3 and NF-κB in HepG2.2.15 cells was enhanced. BM-06 was selected as a TLR3 synergist capable of activating the TLR3/interferon pathway most effective among 4 synthetic dsRNAs. The migration and proliferation were significantly inhibited in treated HepG2.2.15 cells with BM-06 or Sorafenib alone as compared with PBS-sham control (P < 0.01). However, the role of combination BM-06 with Sorafenib was the most prominent. Tumor cell apoptotic rate was increased by BM-06 or combination when compared to PBS or poly(I:C) (P < 0.05). Similarly, in orthotopic HCC SD rats, the effect of the combination was superior to either agent alone on the inhibition of tumor growth and induction of HCC cell apoptosis (P < 0.05).

**Conclusions:**

dsRNA alone was capable of inhibiting the proliferation of HepG2.2.15 cells and tumor growth of orthotopic HCC SD rats, but the effect of combination of dsRNA with sorafenib was more prominent. These findings implicate the potential role of combined use of a dsRNA, a TLR3 synergist, and sorafenib in inhibition of HCC.

## Background

Hepatocellular carcinoma (HCC) is a complex and heterogeneous tumor with several genetic alterations. It is the second leading cause of cancer deaths in man and the sixth in women worldwide [1-3]. An estimated 748,300 new liver cancer cases and 695,900 liver cancer deaths occurred in 2008 [4]. However, mechanisms of initiation and progression of liver cancer have not been elucidated completely. Long-term survival rate remains unsatisfactory due to tumor recurrence and limited response to chemotherapy and radiotherapy [5]. Clinically, 70-90% of HCC cases develop due to a background of cirrhosis or chronic liver inflammation [6]. So far, there is a lack of effective systemic therapy for advanced cases. Only 10–20% of HCC patients in China are able to undergo surgical resection due to poor liver function or advanced disease [7]. In the West, 40% of patients can receive potential curative treatment (resection, transplantation, or local ablation) and 20% are suitable for chemoembolization [8-10]. Therefore, development and identification of novel agents that are able to suppress HCC effectively is imperative for advanced HCC patients. The advent of sorafenib and synthetic dsRNAs increases chemotherapeutic options for these advanced patients.

In the past years, sorafenib, a multi-kinase inhibitor, represents a breakthrough in the management of this neoplasm [11]. It is a bi-aryl urea capable of inhibiting multiple receptors of tyrosine kinases (RTK) and Ser/Thr kinases [12]. These include but are not limited to all isoforms of Raf, all isoforms of vascular endothelial growth factor receptors (VEGFR), and platelet-depedent growth factor receptor (PDGFR)-β. This multifunctional profile lends itself to inhibition of tumors via the Ras/Raf/MEK pathway, activation and proliferation of endothelial cells via VEGFR-2 and the Ras/Raf/MEK pathway, recruitment of pericytes via PDGFR-β (required for vessel stabilization and maturity), recruitment of stabilizing stromal cells to the tumor’s parenchyma, as well as subsequent stimulation of stromal cells through growth factors [12-14]. The above effects of sorafenib are similar to that observed with rastuzumab in breast cancer, bevacizumab in colon cancer, and erlotinib in lung cancer with a decrease in the risk of death in the range of 25%-35% [15-17]. The above evidence that increase the efficacy of molecular targeted therapies for liver cancer has triggered a search for additional molecular agents to further prolong patient survival.

TLR3, a member of the Toll-like receptor (TLR ) family, can recognize double-stranded RNA (dsRNA) from viruses, endogenous dsRNA released from dying cells, or synthetic dsRNA such as polyriboinosinic:polyribocytidylic acid (poly I:C). TLR3 signaling depends solely on the TLR TIR domain which contains the adaptor-inducing IFN-ß (TRIF) adapter protein. This leads to activation of the NF-κB and IRF3 transcription factors, and as a result, induces the antiviral interferon response [18,19]. Furthermore, TRIF itself exhibits proapoptotic activity, suggesting that TLR3 signaling can trigger cell death pathway [20]. Recently, the TLR3 ligand dsRNA has been reported to induce apoptosis in several cell types through multiple pathways. In addition, TLR3 may directly trigger apoptosis in certain cancer cells [21,22]. In addition, TLRs in tumor cells facilitate their evasion from immune surveillance via the suppression of T-cell proliferation and natural killer cell activity, suggesting that TLR signaling in tumor cells is associated with the progression of cancer and evasion of host defenses. Thus, TLRs could be considered as potential therapeutic targets in HCC.

Due to the complexity of genetic aberrations in HCC, single agent often fails to suppress tumor growth completely; therefore, combination of two or more anti-cancer agents would greatly increase therapeutic effects.. In this study, we evaluated the expression of a series of proteins relating to TLR3 signaling pathway, such as NF-κB, caspase 8 survivin, bcl2 and PCNA, affected by dsRNA or sorafenib alone or in combination of both. According to the sequence of TLR3 sensitive virus, 4 dsRNAs were synthesizede, and only one was selected as a TLR3 synergist (BM-06) since it was the most effective to activate TLR3. Our results showed that combination of BM-06 with Sorafenib was superior to either agent alone in the inhibition of tumor growth either in vitro HCC cell lines (HepG2.2.15) or in vivo HCC rat models. Future investigations will be focused on the mechanism of the activated TLR3 in inhibiting HCC, and ultimately, a more effective anti-HCC therapy will be evaluated using a combination use of sorafenib and dsRNA.

## Methods

### Cell culture

Human HCC cell line (HepG2.2.15) producing HBV was purchased from Ruijin Hospital (Shanghai, China). The cells were maintained in a Dulbecco’s modified Eagle’s medium (DMEM) (GibCo BRL, Grand Island, NY, USA) supplemented with 20% fetal bovine serum (FBS), 2 mM L-glutamine, and 100 U/mL penicillin-streptomycin mixture (GibCo BRL, Grand Island, NY, USA) at 37°C and 5% CO_2_ in a humidified chamber.

### Design and syntheses of 4 dsRNA TLR3 synergists

Four dsRNAs were designed and synthesized by Biomics.Co. Ltd (Nantong, China). Their antisense sequences are as follows: BM-06: CCGGCCCCUGAAUGCGGCUAAUC; VEGF-siRNA: GAUCCGCAGACGUGUAAAUdTdT; VEGFR-siRNA: GAGUGUAAAAACAUUUGAAdTdT; short (17nt)-dsRNA: GUCCUACUGAUUGAAGU.

HepG2.2.15 cells were seeded into the wells of a 6-well culture plate and allowed to grow until 80% confluence. Subsequently, these cells were treated with the above 4 different dsRNAs, respectively. (10 μg/ml)After treatment at 37°C for 24 hours, the mRNA and protein expressions of TLR3 and NF-κB in HepG2.2.15 cells were measured by qRT-PCR and Western blot, respectively. The dsRNA that showed the most effective activation against TLR3 /interferon pathway was selected for following interventional treatments.

### Treatments of HepG2.2.15 cell line

HepG2.2.15 cells were incubated with the synthetic dsRNA (BM-06), or sorafenib (Bayer) alone, or BM-06 plus sorafenib. In the present study, poly(I:C) (Invivogen San Diego, USA) and phosphate buffered saline (PBS) were used as a positive and a negative control, respectively, by replacing dsRNA or sorafenib. Sorafenib obtained from Nantong Tomor Hospital in the commercially available form of 200 mg tablets was dissolved in 100% DMSO on the day of treatment. Both dsRNAs and sorafenib were incubated with cells at a concentration of 10 μg/ml for 24 hours in *in vitro* experiments.

### Development of orthotopic HCC SD rat model and drug treatment

Forty male Sprague–Dawley (SD) rats, 4–6 weeks old and weighing 120–160 g, were fed with food containing 0.03% 2-acetylaminofluorene (2-AAF, Sigma), a HCC carcinogen, for 16 weeks in an air-conditioned environment. Thirty-five rats were randomly divided into 5 groups (n = 5/group): dsRNA, sorafenib, Poly I:C, dsRNA plus sorafenib and PBS control. Two of the remaining ten rats were euthanized at each time point of 12, 14, 16 ,18 and 20 weeks, respectively, to decide cellular malignant transformation in the livers. All rats were treated and all procedures were conducted in accordance with the guidelines for experimental animals approved by the Animal Care and Use Committee of Nantong University, P.R. China.

Solublized sorafenib was administered intraperitoneally (i.p.) into HCC rats, once a week, at 20 mg/kg. dsRNA and poly(I:C) were suspended in sterile PBS and injected (i.p.) into rats with HCC, once a week, at 1.0 mg/kg. Administration started at 16 weeks after the rats were fed with 2-AAF, and continued for 6 weeks. At the end of treatments, all treated rats were sacrificed, the liver was collected and weighed. Part of the liver tissue was fixed in 10% formalin for pathological examination and immunohistochemical analysis, and the remaining were stored at −80°C for RNA and protein extraction.

### qRT-PCR

Total RNA was isolated from HepG2.2.15 cells and rat HCC liver tissues using TRIZOL (Invitrogen, Carlsbad, CA). qRT-PCR was performed to evaluate TLR3, NF-κB caspase-8 and IFN-γ using an ABI 7700 Sequence Detection Systerm (Applied Biosystems). caspase-8 and IFN-γ were measured only in rat HCC tissues. Cycling conditions for amplification were: 95°C for 3 min; 35 cycles at 95°C for 45 s, 60°C for 45 s, and 72°C for 30 s; and terminated at 72°C for 7 min. The primer pairs were listed in Table 1. All human gene expression was normalized to glyceraldehyde-3-phosphate dehydrogenase (GAPDH) mRNA copies, and rat gene expression was normalized to β-actin mRNA copies in all samples.

**Table 1:** The primer pairs used in the PCR performing

**Number**	**Name**	**Sequence (5′ → 3′)**
H-NF-κB*	-F	GTAGTCCCCACGCTGCTCTTCTATA
	-R	GGAGCAGGCTATCAGTCAGCGC
H-TLR3*	-F	TCCCAGCCTTACAGAGAAGC
	-R	CCTGTGAGTTCTTGCCCAAT
H-GAPDH*	-F	GAAGGTGAAGGTCGGAGTC
	-R	GAAGATGGTGATGGGATTC
R-TLR3^#^	-F	CGGTCAAGGTGTTCAAGA
	-R	GGATGGTAGAAGCGTGTT
R-NF-κB^#^	-F	TGGCTTCTATTACCTGTA
	-R	TAACGACATATACCATCAG
R- caspase-8^#^	-F	TGAACTATGATGTGAGCAATA
	-R	TTCCGTAGTGTGAAGATG
R-IFN-γ^#^	-F	TCTTCACATCAAAGGAGTCATC
	-R	TGCTGCTGGAGGTCATTA
R-β-actin^#^	-F	TATGGAATCCTGTGGCATC
	-R	GTGTTGGCATAGAGGTCTT

* Primer pairs were designed for human (H) HepG2.2.15 cells; and ^#^ Primer pairs designed for rat (R) HCC tissues.

### Immunofluorescence

Cells were incubated with a rabbit polyclonal anti-NF-κB-p65 antibody (Table 2) at a dilution of 1:100 as the primary antibody. A goat anti-rabbit IgG conjugated with FITC (Table 2) was used as the secondary antibody at a dilution of 1:100. Samples were counterstained with Hoechst 33258 and photographed using a confocal microscope (Olympus, BX51, Japan).

**Table 2:** The antibodies used in immunohistochemical staining and Western blot

**Antibody**	**Producer**	**Applications**	**Working dilutions**	**Positive localization**
TLR3	Abcam	Western blot	1:1000	cytoplasmic
			1:100	
NF-κB p65	Cell Signaling Technology	Western blot Immunofluorescence	1:1000	cytoplasmic
			1:100	nucleus
Lamin B	Santa Cruz Biotechnology,	Western blot	1:100	nucleus
α-tubulin	Santa Cruz Biotechnology,	Western blot		cytoplasmic
Survivin	Santa Cruz Biotechnology	Western blot	1:1000	cytoplasmic
PCNA	Santa Cruz Biotechnology	Western blot	1:1000	nucleus
BCL-2	Santa Cruz Biotechnology	Western blot	1:1000	cytoplasmic
β-actin	Santa Cruz Biotechnology	Western blot	1:2500	
Goat anti-rabbit IgG	Cell Signaling Technology	Western blot Immunohistochemical	1:1000	
			1:100	
Goat anti-rabbit	Multiscience	Immunofluorescence	1:100	
IgG(H + L),FITC				

#### Cell proliferation assay

Cell proliferation was measured using the Cell Counting Kit-8 (CCK-8) (Dojindo, Kumamoto, Japan) assay following manufacturer’s instructions. Briefly, HepG2.2.15 cells were seeded on a 96-well cell culture cluster (Corning Inc., Corning, NY) at a number of 2 × 104/well in a volume of 100 μl, and allowed growing overnight. Next day, CCK-8 reagents were added to each wells under different treatments and incubated at 37°C for 2 hours. Absorbance was measured for quantification on an automated plate reader. Each treatment was conducted in triplicates.

### Flow cytometry assay

Flow cytometry (Beckman Coulter, Fullerton, California, USA) was used to determine the apoptotic rate. The HepG2.2.15 cells treated with the synthetic BM-06, or sorafenib alone, or BM-06 plus sorafenib?? were suspended in a 500 μl binding buffer (Becton Dickinson, USA), incubated with 5 μl Annexin V- FITC/PI (Becton Dickinson, USA) and 5 μl propidium iodide (PI) (Becton Dickinson, USA) for 15 minutes. Phosphatidyl serine translocation to the cell surface serves as an indicator of early apoptotic cells; therefore, annexin V-positive and PI-negative cells were identified as apoptotic cells. The apoptotic rate was determined using Cell Quest software (FCM, Becton Dickinson).

### Cell invasion assay

HepG2.2.15 cells (2 × 10^4^/well) were seeded and incubated in 24-well at 37°C and 5% CO_2_ for 24 h.Transwell chambers (Corning Inc., Corning, NY) were pretreated with DMEM for 30 min. HepG2.2.15 Cells were treated with 2.5% trypsin and suspended in a serum free DMEM medium at a concentration of 1 × 10^6^/ml prior to added into each upper chamber (200 μl), and 600 μl DMEM medium containing 20% FBS with different agents were added into each lower chamber. Subsequently, the transwell chambers were incubated in a 37°C, 5% CO_2_, humidified incubator for 48 h. The cells on the inner surface of the filter membrane (8.0-μmpore size) were removed. The cells on the lower surface of the membrane were stained with crystal violet, and counted in five random fields under a light microscope (200X).

### Hoechst staining

Treated cells were exposed to staining solution containing Hoechst 33258 (1 μg/ml) (Beyotime Institute of Biotechnology, China) at 37°C for 20 min. Cells with chromatin condensation were visualized and photographed using a digital fluorescence microscope (Olympus) at 30 min after addition of the staining solution. Chromatin condensation is the most characteristic feature of apoptosis. Cell apoptotic ratio was obtained by counting the number of apoptotic cells with condensed nuclei amoung all number of cells in six to eight randomly selected areas.

### Nuclear and cytoplasmic extraction, Western blot analysis

Cells were seeded on a 6-well cell culture cluster (Corning Inc.) at a concentration of 5 × 10^4^/well in a volume of 2 ml, and grown overnight. Cells were treated with 10 μg/ml BM-06 or poly(I:C) or 10 μl PBS as control and incubated for 24 h at 37°C. Briefy, cell pellets from a culture were incubated in a hypotonic buffer [10 mM HEPES (pH 7.2), 10 mM KCl, 1.5 mM MgCl2, 0.1 mM EDTA, 20 mM NaF, 100 μM Na3VO4, and protease inhibitor mixture] for 30 min at 4°C on a rocking platform. Cells were homogenized (Dounce, 30 strokes), and their nuclei were pelleted by centrifugation (10 min × 14,000 rcf, 4°C). The supernatant was saved as the cytosolic fraction, and nuclear pellets were incubated in nuclear lysis buffer [10 mM Tris–HCl (pH 7.5), 150 mM NaCl, 5 mM EDTA, and 1% Triton X-100] for 1 h at 4°C on a rocking platform. The nuclear fraction was collected by centrifugation (10 min × 14,000 rcf, 4°C).

Prior to immunoblotting, the rat HCC tissues were homogenized inlysate buffer containing protease inhibitors and then pelleted via centrifugation at 13,000 g at 4°C. The protein concentration in supernatants was measured and 100 μg of proteins were loaded in each well of 10% SDS-PAGE gels for electrophoresis prior to electroblotting proteins onto polyvinylidene difluoride (PVDF) membrane (Immbilon, Millipore). The membrane was incubated with anti-phospho-NF-κB p65, anti-TLR3, PCNA, Survivin and BCL-2 (Table 2) primary antibodies at 4°C overnight following blockading non-specific binding sites in 5% non-fat milk in TBST (Tris-buffered saline containing 0.1% Tween-20). The membranes were washed 3 times in TBST for 5 minutes and subsequently incubated with secondary antibody for 2 hours at room temperature. The bands on the membrane were displayed on the film using a chemiluminescence system (Pierce, Rockford, IL, USA). The bands on the film was scanned and measured for their density using Image Quant software (Molecular Dynamics, Sunnyvale, CA, USA). The ratios of NF- κB or TLR3 to β-actin were obtained.

### Hematoxylin and eosin (HE) staining

After harvest, rat HCC tissues were formalin-fixed, paraffin-embedded, and sections (4 μm thick) were prepared for standard hematoxylin/eosin (H&E) and immunohistochemical staining. The changes in histology were assessed under a light microscope.

### TUNEL(Terminal deoxynucleotidyl transferase-mediated dUTP nick-end-labeling)detected apoptosis

TUNEL detection kit (Promega, USA) were employed for the detection of neuronal apoptosis. In brief, paraffin-embedded sections were deparaffinized and dehydrated. After washing in PBS, sections were treated with 20 μg/mL Proteinase K for 20 min. After washing in PBS thrice (3 min for each), sections were rinsed with 0.3% Triton X-100 for 10 min followed by washing in PBS. These sections were incubated with TUNEL reaction mixture at 37°C for 1 h. Following washing in PBS thrice (3 min for each), sections were treated with HRP conjugated streptavidin (1:200; Beijing Zhongshan Biotech Co., Ltd) at 37°C for 30 min. After washing in PBS thrice (3 min for each), sections were treated with 0.04% DAB and 0.03% H2O2 at room temperature for visualization for 8–12 min. After washing in water, counterstaining was done with hematoxylin followed by mounting with resin. In the negative control, TUNEL reaction mixture was replaced with PBS. The positive control sections were pre-treated with DNase I for 10 min followed by TUNEL staining. Cells with blue granules in the nucleus were regarded as positive for TUNEL. A total of 100 cells were counted at a high magnification, and the percentage of TUNEL positive cells was calculated.

### Statistical analysis

Statistical analysis was performed using SPSS 17.0 for Windows. The data were expressed as a mean ± SD. Differences between groups were evaluated with ANOVA or factorial design ANOVA and considered statistically significant when P < 0.05. Nodules size was quantified using Histolab 5.8 software (Microvision Instruments).

## Results

### Identification of the most effective dsRNAs activating TLR3

qRT-PCR results showed that both TLR3 and NF-κB were expressed in HepG2.2.15 cells. Five dsRNAs, VEGFsiRNA (si-VEGF), VEGFRsiRNA (si-VEGFR), 17ntdsRNA (17 bp), BM-06 (23 bp)and poly(I:C), were chosen to identify the most effective RNA nucleic acid in activation of TLR3 (Figure 1). qRT-PCR analyses showed that all five dsRNAs resulted in increases in mRNA expression of both TLR3 and NF-κB in HepG2.2.15 cells, but dsRNA BM-06 revealed most effective in the activation of TLR3; therefore, it was selected for further studies in the following experiments. Since BM-06 or poly(I:C) bound to TLR3 will activate NF-κB and might regulate the nuclear-cytoplasmic shuttling, NF-κB activity was checked by immunofluorescence after treating HepG2.2.15 with BM-06 or poly(I:C). Immunofluorescence analysis showed BM-06 or poly(I:C) treated HepG2.2.15 cells which expressed NF-κB levels predominantly in the nuclear fraction but fewer signals in the cytoplasm (Figure 2A). To corroborate these findings, we then tested the expression of endogenous NF-κB of HepG2.2.15 cells under treatment with BM-06 or poly(I:C). Western blot analysis showed BM-06 or poly(I:C) treated HepG2.2.15 cells which expressed NF-κB levels predominantly in the nuclear fraction but fewer signals in the cytoplasm (Figure 2B).

**Figure 1:** **TLR3 and NF-κB mRNA expressions.** The expressions of TLR3 and NF-κB were determined by RT-qPCR in HepG2.2.15 cells treated with five different dsRNAs**.** The values in the figure are normalized to PBS treatment (1.00). *, p < 0.05 compared to the PBS control group; #, p < 0.05 compared to the BM-06 group.

**Figure 2:** **Expression of NF-κB-p65 in HepG2.2.15 cells. A**: Detection of NF-κB-p65 expression in cells by immunofluorescence staining. NF-κB p65 (green) was expressed in HepG2.2.15 cells. BM-06 and poly(I:C) induced TLR3-activated HepG2.2.15 cells expressing NF-κB levels predominating in the nucleus fraction. The effect of BM-06 was better than the poly(I:C). **B**: Western blot analysis of dsRNA induced TLR3-activated HepG2.2.15 cells expressing NF-κB levels predominating in the cytoplasmic fraction. Cytoplasmic and nuclear fractions were assayed for NF-κB protein (α-tubulin, cytoplasmic marker; lamin B, nuclear marker).

### Effect of combined use of BM-06 and sorafenib on suppression of cell proliferation and invasion, and induction of apoptosis

To determine whether synthetic BM-06 was able to affect the proliferation of HepG2.2.15 cells, a CCK-8 assaywas performed on cells for 24 h, 48 h and 72 h (Figure 3A). The results showed that the proliferative capacity of HepG2.2.15 cells was significantly reduced by BM-06, sorefenib, poly(I:C) alone and BM-06 plus sorafenib compared with the PBS control (P < 0.01; P < 0.01; P < 0.05; P < 0.01, respectively), but the effect of combination was the most significant among treated groups (p < 0.05).

**Figure 3:** **Proliferative capacity and apoptotic cells were observed in all treated groups. A**: The effects of BM-06 plus sorafenib group were the most significant. **A**: Effect of 4 dsRNAs on proliferation of HepG2.2.15 cells. Growth curve of HepG2.2.15 cells was shown for each group. The proliferation was assayed in triplicates at 24 h, 48 h, and 72 h post-treatment using CCK-8 kits. (*, *P* **< 0.05 vs control group;#, *P*** **< 0.05 vs BM-06 + sorafenib group) B**: Apoptotic rates were measured in the treated HepG2.2.15 cells using a FACS analysis after Annexin-V-PI staining. Percentages of apoptotic cells included both early- and late-stage apoptosis (AV+/PI- and AV+/PI+). Increased rates of apoptosis in the treated groups were calculated relative to the PBS control. **C**: Apoptotic cells were observed in Hoechst nuclear staining (X200). **D**: Migrating cells were observed in a Transwell chambers assay (X100).

Whether inhibition of cell proliferation by BM-06 resulted from induction of apoptosis, and synergized by sorafenib. The annexin V-FITC/PI double staining and Hoechst nuclear staining were used to display apoptotic cells. Typical apoptotic feature with Hoechst nuclear staining was showed in Figure 2C. The results of flow cytometry showed the percentage of annexin V-positive/ PI-negative cells was significantly increased in all treated groups (Figure 3B). The apoptotic rates in BM-06, sorafenib, poly(I:C) alone and BM-06 plus sorafenib groups were 20.89%, 23.18%, 19.94% and 26.14%, respectively, compared to as PBS control (13.05%) (all P < 0.01), suggesting that all of these agents resulted in decreased cell viability and increased cell apoptosis. Expectedly, apoptosis rate in the combination group was higher over any of the other treated groups (P < 0.05).

The invasion ability of HepG2.2.15 cells treated with BM-06, poly(I:C), sorafenib, BM-06 plus sorafenib was assessed using a chamber precoated with Matrigel. After 48 h incubation, the cells migrating through Matrigel were counted. A significant decrease was found in the treated groups with BM-06 (74 ± 08), sorafenib (56 ± 23), poly(I:C) (79 ± 04) or BM-06 plus sorafenib (33 ± 16) as compared to the PBS control (140 ± 11) (all P < 0.01), but migrating cells were reduced mostsignificantly in the BM-06 plus sorafenib group(P < 0.01) (Figure 3D).

### Growth inhibition by co-administration of BM-06 and sorafenib in orthotopic SD HCC rat

After fed with 2-AAF for 14 weeks, the liver tissue were observed after the rats were put to death and the tumor nodules were marked by the yellow box. All rats were carcinogenic success (Figure 4A). All SD rats revealed clear histological malignant transformation in the liver (Figure 4B). BM-06, sorafenib, poly(I:C) or BM-06 plus sorafenib was administered into rats for 6 weeks at 2 more weeks after 14 week of feedingwith 2-AAF. The treated rats were sacrificed, and tumor size is mainly compared by liver/body weight ratio of the mice (Figure 4A,C). The results showed that the tumor volumes of the HCC rats treated with BM-06, sorafenib, poly(I:C) or BM-06 plus sorafenib were all significantly reduced when compared with PBS controls (all p < 0.05). Comparison among treated groups showed that the effect of BM-06 plus sorafenib was most prominent on reducing tumor volume (p < 0.05). None of the other organs displayed pathological lesions, suggesting that these agents had no obvious cytotoxic effects on these organs of the experimental rats.

**Figure 4:** **The effects of dsRNAs on HCC of rats after 2-2AAF administration. A**:The liver tissue were observed after the rats were put to death and the tumor nodules were marked by the yellow box. **B**: Histological sections showing malignant features in livers of orthotopic SD rat after fed with 2-AAF(X200). **C**: The ratios of tumors to body weights . *, p < 0.05 versus the PBS control group; #, p < 0.05 versus the BM-06 plus sorafenib group.

In addition, as shown in Figure 5, expression ratios of PCNA (a proliferation marker), survivin and bcl-2 (both anti-apoptosis markers) in tumor cells of the control animals were greater than those of treated rats with BM-06, sorafenib, poly(I:C) and BM-06 plus sorafenib groups. As expected, combination resulted in more significant decreases in the expression of PCNA, survivin and bcl-2 (P < 0.05).

**Figure 5:** **Detection of the expression of PCNA, survivin and bcl-2 by western blot.** Expressions of PCNA, survivin and bcl-2 in orthotopic SD rat HCC . *, p < 0.05 compared to the PBS control group; #, p < 0.05 compared to the BM-06 plus sorafenib group.

Furthermore , the results of TUNEL detection shown that the apoptosis index in tumor cells of the control animals (14.39%) were obviously lower than those of treated rats with BM-06, sorafenib, poly(I:C) and BM-06 plus sorafenib groups (83.61%, 84.38%, 76.53% and 96.42%), respectively (P < 0.05). And that combination resulted in more significant increases the apoptosis index in tumor cells (Figure 6).

**Figure 6:** **TUNEL detected apoptosis in experimental groups.** Apoptotic nuclei were stained in brownish yellow, while normal nuclei were stained in blue. (hybridization in situ × 400).

As shown in Figure 7A, the RT-qPCR analyses showed that the mRNA expression of TLR3, NF-κB, caspase-8 and IFN-γ in liver tumors of the HCC rats was all significantly up-regulated by BM-06, poly I:C or BM-06 plus sorafenib. Western Blot assay revealed that increases in protein expression of TLR3 and NF-κB were observed in 3 groups treated with BM-06, poly I:C or BM-06 plus sorafenib (Figure 7B) in comparison with the PBS control (P < 0.05). In contrast, no difference in the expressions of TLR3, NF-κB and IFN-γ was present in sorafenib alone versus PBS , but an increased mRNA expression of caspase-8 was found by sorafenib alone.

**Figure 7:** **The expression of TLR3, NF-κB, casepase-8 and IFN-γ in the tumors. (A)** The mRNA levels of TLR3, NF-κB, casepase-8 and IFN-γ; **(B)** TLR3 and NF-κB protein levels in liver tumors determined by Western Blot. Densitometric analyses of TLR3 and NF-κB proteins relative to β-actin. Values are normalized to control cells (1.00). *, p < 0.05 compared to the PBS control group; #, p < 0.05 compared to BM-06 plus sprafenib group; **(C)** Western blot showing the bands of TLR3 and IFN-γ proteins.

## Discussion

Molecular targeted therapies have created an encouraging trend in the management of cancer. Sorafenib is a multikinase inhibitor with a reported activity against Raf-1, B-Raf, VEGFR2, PDGFR, c-Kit receptors, and other receptors tyrosine kinases and serine threonine kinases [23]. Sorafenib has been used in patients with advanced HCC and also for those progressing after local therapies.Although preclinical studies showed potent activity of sorafenib in decreasing HCC cell viability and inducing apoptosis, it also has anti-angiogenic effect in vitro and in vivo, and antitumor activity in xenograft models., This study was aim at improving its efficacy by combining with other new drugs and capable of suppressing tumors by involving in other pathways.

TLR3 is a member of TLR family of innate immune response receptors implicated in the initial host defense against bacteria and viruses through the recognition of specific pathogen-associated molecular ligands, and stimulation of intracellular signaling, leading to the secretion of inflammatory cytokines. Preclinical studies have shown that dsRNAs as a TLR synergist can boost innate immunity, augment antibody-dependent effect or functions, and enhance adaptive immune responses [24-26]. TLR3 may directly trigger apoptosis in certain cancer cells. Therefore, TLR3 when activated by dsRNAs may be a potential target for certain tumor treatment [27]. Further studies will be conducted on the mechanisms for dsRNA alone or in combination with sorafenib in inhibiting tumors.

Several studies have demonstrated that TLR3 was expressed on cell surface and in the cytoplasm of Kupffer cells, hepatic stellate cells, hepatic immune cells, liver sinusoidal endothelial cells, and normal and tumor hepatocytes, [28-30]. Although some cancer cells, such as colonic adenocarcinoma, lung cancer, breast cancer and melanoma, were also reported to express TLR3, the exact roles of TLR3 in these cancer cells have yet to be elucidated [21,31-33]. The TLR3 inflammatory pathway leads to the NF-κB activation; whereas NF-κB is shown to induce pro–IL-1β expression in hepatocytes, which is then activated by caspase-8, an apoptotic pathway mediated by Rip3 [34], leading to hepatocyte death. Several studies have shown that in human hepatoma cell lines, unlike white blood cells, TLR3 signaling is skewed towards the apoptotic pathway [35]. In the present study, both HepG2.2.15 cells and rat tumor tissue were able to express TLR3 and NF-κB. We selected BM-06 dsRNA as a TLR3 synergist to stimulate TLR3 signaling, which leads to the activation of NF-κB and upregulation of caspase-8 and IFN-γ, thus initiating the TLR3 mediating inflammatory and apoptotic pathways.

Apoptosis is one of the mechanisms leading to cell death when cells have sustained damage to their DNA or cytoskeleton [36]. After dsRNA treatment, HepG2.2.15 cell apoptosis was enhanced and activity was decreased. In HCC rats treated with dsRNA, especially combination with sorafenib, the increase in the expressions of TLR3, NF-κB, caspase-8 and IFN-γ resulted in down-regulation of survivin, bcl-2 and PCNA, which indicates increased apoptosis and inhibition of tumor growth. TUNEL assay confirmed that BM-06 can cause the HepG2.2.15 cell apoptosis as well as sorafenib, the role of combination BM-06 with Sorafenib was the most prominent and had better antitumor action. Similarly, Khvalevsky [34] discoverd that during the initial regenerating phase following partial hepatectomy, TLR3 signaling was induced in hepatocytes, leading to activation of NF-κB and caspase-8, and an increase in Rip3 protein levels. Upon activation, caspase-8 cleaves effector caspases, which leads to cell death by initiating apoptotic program. Yoneda et al. [37] found cytoplasmic stimulation by transfected Poly I:C significantly induced apoptosis accompanied by the down-regulation of anti-apoptotic protein. Our findings suggest that HCC cells were able to respond to these dsRNAs, thus apoptosis was induced, and proliferationand invasion were suppressed via binding TLR3 on the HCC cell surface. TLR3-mediated signaling leads to the activation of NF-κB and IRF-3 and expression of inflammatory associated with genes, including interferons [38]. In this study, a level of INF-γ in the liver tumors was significantly increased in the rat treated with BM-06. INF-γ has been identified as an inhibitor of endothelial cell proliferation and a potent suppressor of tumor-associated neovascularization. Similarly, Mathieu studies showed [39] that treatment of HCC mice with poly(I:C) resulted in suppression of vasculature remodeling and liver tumor growth. These effects might result from the activation of endothelial cellsurface TLR3 and subsequent up-regulation of INF-γ and interleukin-12. However, their investigations showed that the INF-γ in mouse HCC liver extracts was most likely released by circulating or resident immune cells. Recent evidence indicates that TLR3 may contribute to suppression of tumor growth through the interferon-dependent activation of NK cells and expansion of Treg lymphocytes [40]. In short, the mechanism by which dsRNA activates TLR3 is very complex and, further studies will be conducted.

In this study, although the effect of BM-06 alone is less significant than that of sorafenib alone in inhibition of HCC proliferation, it is able to augment the role of sorafenib when combined with it. In addition, dsRNA could play a role in inhibition of HCC through additional pathways, in which sorafenib might be ineffective that disrupts more pathways in the complex tumor microenvironment. Therefore, application of combination of BM-06 with sorafenib would be an ideal option in treatment of patients with cancers because such a combination can simultaneously block signaling through the sorafenib MEK or synergize TLR3 signaling. In addition, the combination of both agents could attenuate systemic toxicity in animals. The optimal length of dsRNA that can activate TLR3 in vivo is still unclear. In suppressing tumor vasculature remodeling, unlike 21- and 23-nucleotide Luc siRNA, 7-, 13-, 16-, or 19-nucleotide versions failed to suppress choroidal neovascularization (CNV) [41]. Thissuggests that RNAs with a length at least 21 nucleotides are required to activate TLR3, whereas longer dsRNA could be more cytotoxic. In the present study, BM-06, a length of 25 nucleotide, was able to activate TLR3. Similarly, 17 nucleotide dsRNA also activated TLR3, although the effect of shorter dsRNA (17 nucleotide) was less than that of 25 nucleotide dsRNA (BM-06). BM-06 was superior to poly(I:C) in inhibiting the proliferation and promoting apoptosis of HepG2.2.15 cells, especially in combination with sorafenib. These results show that stimulation of TLR3 by dsRNA may be sequence length sensitity. Further investigations will be focused on selection of more effective TLR3 dsRNAs and exploration of more exact mechanisms in activation of TLR3 in prevention of tumors.

As therapeutic agents, synthetic dsRNAs provide some advantages over small inference RNA (siRNA), including possibility for chemicalconformation that could increase their efficiency and attenuate off target suppression effects. Since synthetic siRNAs must be transfected into the target cells through a vector, such as Lipofectamine™ 2000 reagent, they always exhibit cytotoxicity, which may limit their use in clinic. TLR3 ligand dsRNA is able to inhibit tumor growth; therefore, it could be used for adjuvant therapy in prevention of HCC.

## Conclusion

dsRNA alone was capable of inhibiting the proliferation of HepG2.2.15 cells and tumor growth of orthotopic HCC SD rats, but the effect of combination of dsRNA with sorafenib was more prominent. Combination therapy can target multiple receptors and signaling pathways. Many of these combinations have been shown in preclinical studies to have synergistic effect and may block proposed resistant pathways.

## Competing interest

The authors declare that they have no competing interests.

## Author’s contributions

LC conception and design of research; YYX carried out the molecular genetic studies, participated in the sequence alignment and drafted the manuscript. YYX, JQ, YXZ and YYZ analyzed data; YYX interpreted results of experiments; YYX and GLW prepared Figures; LC and YYX edited and revised manuscript; YYX approved final version of manuscript; YYX, JMZ and YZW performed experiments. All authors read and approved the final manuscript.

## Pre-publication history

The pre-publication history for this paper can be accessed here:

http://www.biomedcentral.com/1471-2407/13/527/prepub
